# Machine learning-based transcriptome analysis of lipid metabolism biomarkers for the survival prediction in hepatocellular carcinoma

**DOI:** 10.3389/fgene.2022.1005271

**Published:** 2022-09-28

**Authors:** Ronghong Xiong, Hui Wang, Ying Li, Jingpeng Zheng, Yating Cheng, Shunfang Liu, Guohua Yang

**Affiliations:** ^1^ Second Clinical College of Wuhan University, Zhongnan Hospital of Wuhan University, Wuhan, China; ^2^ Department of Medical Genetics, School of Basic Medical Science, Demonstration Center for Experimental Basic Medicine Education, Wuhan University, Wuhan, China; ^3^ Department of Oncology, Tongji Hospital, Tongji Medical College, Huazhong University of Science and Technology, Wuhan, China

**Keywords:** lipid metabolism, hepatocellular carcinoma, machine learning, prognostic risk model, biomarkers

## Abstract

Hepatocellular carcinoma (HCC) is the most common primary malignancy of the liver with a very high fatality rate. Our goal in this study is to find a reliable lipid metabolism-related signature associated with prognostic significance for HCC. In this study, HCC lipid metabolism-related molecular subtype analysis was conducted based on the 243 lipid metabolism genes collected from the Molecular Signatures Database. Several significant disparities in prognosis, clinicopathological characteristics, and immune and ferroptosis-related status were found across the three subtypes, especially between C1 and C3 subgroups. Differential expression analysis yielded 57 differentially expressed genes (DEGs) between C1 and C3 subtypes. GO and KEGG analysis was employed for functional annotation. Three of 21 prognostic DEGs (CXCL8, SLC10A1, and ADH4) were finally selected through machine-learning-based discovery and validation strategy. The risk score = (0.103) × expression value of CXCL8 + (−0.0333) × expression value of SLC10A1 + (−0.0812) × expression value of ADH4. We used these three to construct a HCC prognostic risk model, which stratified the patients of the validation cohort into two risk subtypes with significantly different overall survival. Our work provides possible significance of the lipid metabolism-associated model in stratifying patient prognosis and its feasibility to guide therapeutic selection.

## Introduction

As a leading cause of cancer-related death worldwide, hepatocellular carcinoma (HCC) is the most prevalent type of primary liver malignancy (Balogh et al., 2016). Patients with HCC have a wide range in overall survival rates from region to region (Sung et al., 2021), with a 5-years survival rate of only 18% in the United States (Jemal et al., 2017). The most major risk factors for the development of HCC are chronic liver disease and cirrhosis, with viral hepatitis and excessive alcohol consumption being the primary well-known etiologies (Bruix et al., 2004). Therefore, it is vital and urgent to identify the prognostic value of novel markers that can aid in selecting patients who will benefit from patient-specific strategies.

The tumor microenvironment (TME) facilitates tumor metastasis, proliferation, and survival, which leads to abnormal metabolisms for tumor cells and those adjacent stromal cells. The TME in HCC might indicate a variety of metabolic disturbances, with lipid metabolic anomaly being a fresh subject that has sparked a lot of interest in recent years (Beloribi-Djefaflia et al., 2016). Lipid metabolic disturbance, particularly for fatty acid (FA) metabolism, is associated with altered lipid-metabolizing enzyme expression and activity due to aberrantly activated oncogenic signaling pathways (Hu et al., 2020). Lipid metabolism has been increasingly recognized as a critical phenomenon of metabolic rewiring within immune cells and cancer cells, which may be involved in the development of HCC. Furthermore, evidence from various solid tumor research suggests that tumor immune-metabolic reprogramming is significant, and it has been designated as a new critical subject for future HCC studies (Zhang et al., 2018). According to prior research, immune cells play an important role in the TME of HCC, and aberrant lipid metabolism may have a major impact on their activities and recruitment (Gajewski et al., 2013). Although growing studies have explored the genetic, cellular, and environmental mechanisms involved in the development of tumors (Chen et al., 2020; Zhang et al., 2020; Cao et al., 2021a; Zhong et al., 2021), clinicians currently have few choices for slowing HCC progression and extending patients’ lives. Therefore, integrated lipid metabolism and liver cancer progression to build an effective prediction model is needed and is the focus of this investigation.

In this study, our goal is to identify a robust lipid metabolism-related signature associated with the HCC microenvironment to improve the prognostic prediction of HCC patients. Genes related to energy metabolism were collected from the Molecular Signatures Database. Gene expression data from The Cancer Genome Atlas (TCGA) were used in constructing HCC molecular subtypes based on genes related to energy metabolism. The relationship between molecular subtypes and prognosis was further evaluated. After differential expression analysis and machine-learning-based selection, three lipid metabolism-driven signatures were chosen from the 576 differentially expressed genes (DEGs) for establishing a prognostic risk model. Then, we validated the risk model, which may be used to assess the prognosis of HCC patients. Overall, this 3-signature prognostic risk model (CXCL8, SERPINC1, and ADH4) we built can be used as an independent prognostic evaluation index for HCC patients.

## Materials and methods

### Data collection and preprocessing

RNA-sequencing expression (level 3) profiles and corresponding clinical information for 371 HCC as well as 50 healthy subjects were derived from the TCGA dataset (https://portal.gdc.com). The raw data were preprocessed with the criteria which have been described elsewhere (Cao et al., 2020; Mao et al., 2020; Cao et al., 2021b; Mao et al., 2021). A total of 243 lipid metabolism-associated genes were gathered based on the Molecular Signatures Database v7.5.1 (c2: curated gene sets), including Fatty acid metabolism M699, Glycerophospholipid metabolism M9131, Glycerolipid metabolism M15902, Sphingolipid metabolism M15955, Ether lipid metabolism M2130, Glycosphingolipid biosynthesis-ganglio series M8535, Biosynthesis of unsaturated FAs M11673, Glycosphingolipid biosynthesis-globo series M12899, Glycosphingolipid biosynthesis-lacto, and neolacto series M17377 (http://www.broadinstitute.org/gsea/msigdb/index.jsp).

### Identification and validation of the lipid-related subtypes

Consensus clustering was applied to identify a robust cluster of HCC patients based on the expression profile of The Cancer Genome Atlas Liver Hepatocellular Carcinoma (TCGA-LIHC) data (Cao et al., 2020). The 1,000 bootstraps with 80% item resampling and a range of K from 2 to 10 were selected for clustering analysis. Partition around the medoids classifier was trained in the discovery cohort. By calculating the in-group proportion and Euclidean correlation in the centroid of gene module scores, we quantitatively acquired and verified the consistency of immune subtypes among populations. The expression value for lipid metabolism-associated gene within each subtype was used for Principal component analysis (PCA) by the “prcomp” function in R.

### Immune status and ferroptosis-related estimation

We used the CIBERSORT method (Chen et al., 2018) to assess the immune composition of a tumor biopsy and get reliable results of immune score evaluation. The relative abundance enrichment score of 22 Tumor infiltrating leukocytes (TILs) was measured and standardized from 0 to 1. Moreover, potential immune checkpoint blockade (ICB) response was predicted with Tumor Immune Dysfunction and Exclusion (TIDE) algorithm (Jiang et al., 2018). Twenty-four Ferroptosis-related genes were collected from the previous study (Liu et al., 2020). The expression distribution of ferroptosis-related mRNA in tumor and normal tissues was implemented by the R program v4.0.3.

### DEG identification and functional enrichment analysis

The differentially expressed genes (DEGs) of the subtypes were identified using the “limma” algorithm for subsequent analyses (FDR adjusted *p*-value < 0.05 and |log_2_FC| > 3; FC, fold change, FDR, False Discovery Rate) (Ritchie et al., 2015). Afterward, Gene Ontology (GO) terms and Kyoto Encyclopedia of Genes and Genomes (KEGG) functional enrichment analyses were conducted based on the DEGs (Wu et al., 2021). The GO terms and KEGG pathways with a *p*-value of < 0.05 were considered significantly enriched function annotations.

### Development and validation of the prognostic signature

To identify overall survival (OS)-related genes from DEGs and detect lipid metabolism-driven prognostic signature (LMSig), we randomly divided the mRNA expression profile of 371 HCC patients into two parts as the discovery (186 samples) and validation data (185 samples). Then, machine-learning-based variable selection was carried out on the discovery data using likelihood-based boosting in the Cox model as implemented in the R package “CoxBoost” [30]. The machine-learning algorithm has been as described previously in detail (Hou et al., 2021). For the CoxBoost model, the number of boosting iterations was then optimized through cross-validation after the optimal penalty had been determined through ten cross-validations using the R package “CoxBoost” (De Bin, 2016). The CoxBoost algorithm was used to automatically estimate the optimal number of LMSig.

In addition, we used the validation data to further confirm the relationship between LMSigs and clinical/prognostic features of HCC. The *p*-values and hazard ratio (HR) with 95% confidence interval (CI) were generated by log-rank tests and univariate cox proportional hazards regression in Kaplan–Meier curves analysis using the R package “survival” (Therneau and Lumley, 2015; Zhou et al., 2019). The concordance statistic (C-statistic index) was used to measure the goodness of fit of the prognostic model. The time-dependent receiver operating characteristic (ROC) curve was used to appraise the prognostic performance of the risk model for survival prediction, and the area under the ROC curve (AUC) values were calculated with the R package “timeROC” (Blanche and Blanche, 2019).

### Statistical analysis

The statistical difference between the two groups was compared through the Wilcox test, the significant difference between the three groups was tested with the Kruskal–Wallis test. All statistical tests were two-sided, *p*-value < 0.05 was considered statistically significant. All the data were processed and analyzed by R program v4.0.3.

## Results

### Lipid metabolic molecular subtypes of HCC identification

An expression profile of 243 common lipid-related genes in 371 HCC patients from the TCGA database was used to implement the consensus clustering. The analysis clustered the patients with HCC into three subgroups C1, C2, and C3 (Figure 1A). These three conceivable subclusters were respectively distinguished *via* first and second principal components (PCs) (Figure 1B). As shown in Figure 1C, the expression levels of lipid metabolism-related genes seem to differ among the three subtypes. Prognosis signature among them was further analyzed. The Kaplan–Meier method was used to investigate the overall (OS) of the three subgroups, and we observed that the patients in the C3 subtype had the worst prognosis, while the C2 subgroup had significantly best OS (Figure 1D, *p*-value = 0.0043).

**FIGURE 1:** Identification of potential lipid metabolism-related subtypes of HCC. **(A)** Consistency of clustering results in the heatmap (k = 3), rows and columns represent samples, the different colors represent different types. **(B)** PCA analysis of different subgroups with PC1 and PC2. **(C)** The expression heatmap of lipid metabolism-related genes in three subgroups, red represents high expression, and blue represents low expression. **(D)** Kaplan–Meier survival analysis of the different groups of samples from TCGA dataset, comparison among different groups was made by log-rank test. HR (95% Cl), the median survival time for different groups.

### Clinicopathological and immune infiltration characteristics in three subgroups

The clinicopathological characteristics of the three subtypes were then compared. Tumor T stage, Gleason grade, and type of treatment among subtypes reached statistical significance (Figure 2A). The results manifested that those patients diagnosed with differential T stage and grade were clustered unevenly. T3 stage and G3 accounted for the major proportion of C3 while T1 and G2 were in the majority in C1 (Figure 2A).

**FIGURE 2:** The distribution of clinical and immune characteristics in the samples from different groups. **(A)** Distribution of clinical characteristics across C1-C3 HCC patients. Association between three different subtypes and CIBERSORT immune infiltration **(B)**, ICPs **(C)**, and TIDE score **(D)**. Asterisks (*) stand for significance levels. * represents *p* < 0.05, ** represents *p* < 0.01,*** represents *p* < 0.001.

The results of CIBERSORT showed significant differences in infiltrating immune cell types between the three subgroups. There were more abundant proportions of T cell CD8+and T cell regulatory (Tregs) in the C1 subgroup than in the C3 subgroup. On the other hand, Macrophage M0 was significantly enriched in C3 compared with C1 (*p*-value < 0.05; Figure 2B). Moreover, eight ICPs-associated genes were differentially expressed among C1-3. C3 showed significant upregulation of CD274, CTLA4, HAVCR2, PDCD1, PDCD1LG2, TIGIT, and SIGLEC15, while these genes were down-expressed separately in the C1 tumors (Figure 2C).

To predict the ICB response of identified HCC subtypes, the TIDE score was calculated. The findings showed that the TIDE score was significantly lower in the C1 subtype than in the C3 subtype (Kruskal–Wallis test, *p*-value = 4.9 × 10^−11^; Figure 2D). These discoveries suggested that patients of the C1 subtype may be more sensitive to ICB therapy as judged by the TIDE score.

### Ferroptosis-related estimation among three distinct subgroups

Ferroptosis is known as an iron-dependent form of regulated cell death (RCD) triggered by lipid peroxidation accumulation (Aguilera et al., 2021). Recently, triggering ferroptosis has emerged as a promising therapeutic option for inducing cancer cell death, particularly for malignancies that are resistant to traditional therapies (Liang et al., 2019). In our study, the comprehensive landscapes of ferroptosis-related gene interactions, connections, and their prognostic significance for HCC patients in three subgroups were depicted, respectively (Figure 3A). We found that ferroptosis-related genes in distinct subgroups presented a remarkably different correlation in expression. The expression of each ferroptosis-related gene also differed insignificantly among the three lipid subtypes. As shown in Figure 3B, the expression levels of CDKN1A, HSPA5, EMC2, SLC7A11, NFE2L2, FANCD2, SLC1A5, CS, and CARS1 were highly accumulated in C3 compared to C1 subgroups.

**FIGURE 3:** Ferroptosis-related Estimation in three subgroups. **(A)** The circles represent the ferroptosis-related mRNA, and the line represents the relationship between genes. Red represents positive correlation whereas blue represents negative correlation. The thicker the line, the higher the correlation coefficient. The larger the circle the smaller the log-rank *p* value. Different colors of circles represent different types of clusters. **(B)** The expression distribution of ferroptosis-related mRNA in tumor tissues and normal tissues. Asterisks (*) stand for significance levels. * represents *p* < 0.05, ** represents *p* < 0.01, and *** represents *p* < 0.001.

### DEG identification and functional analysis

Transcriptome differential expression was performed between C1 and C3 subgroups of HCC patients according to the above difference among them. Fifty-seven genes were identified as DEGs at FDR < 0.05 and log_2_FC > 3, of which 27 DEGs were up-regulated, and 30 DEGs were down-regulated (Figures 4A,B). Then, GO functional and KEGG pathway enrichment analyses were performed. The results of KEGG analysis demonstrated that up-regulated DEGs majorly participated in complement and coagulation cascades, cholesterol metabolism, fatty acid degradation, and bile secretion (Figure 4C). Meanwhile, down-regulated DEGs were involved in Hepatitis B, proteoglycans in cancer, and the PI3K−Akt signaling pathway. GO analysis revealed that these DEGs were mostly enriched in steroid metabolic process, terpenoid metabolic process (up-regulated DEGs), and regulation of small GTPase (down-regulated DEGs), which were related to lipid metabolism (Figure 4C).

**FIGURE 4:** DEGs Identification and functional analysis between C1 and C3. **(A)** The volcano plot and heatmap **(B)** of differentially expressed gene analysis between C1 and C3. Red represents up regulation whereas blue represents down regulation. **(C)** GO and KEGG enrichment analysis of up- and down-regulated DEGs.

### Establishing a prognostic risk model

Integrated the differential gene expression and patient survival data from the TCGA cohort, we screened DEGs to discover the feasibility and reliability of a prognostic signature for HCC. Among all 57 DEGs, 21 DEGs were associated with the OS of HCC patients (*p*-value < 0.05). Subsequently, a boosting machine learning algorithm was performed for signature selection from these 21 DEGs and identified three lipid metabolism-driven signatures (3LMSig). Then, the 3LMSig was transformed into a risk scoring model by linear combination of the expression of the 3LMSig as follows: risk score of 3LMSig = (0.103) × expression value of CXCL8 + (−0.0333) × expression value of SLC10A1 + (−0.0812) × expression value of ADH4. Among them, the expression value of CXCL8 was linked positively to HCC risk score, while the expression value of SERPINC1 and ADH4 showed a negative relationship with HCC risk score.

According to the risk score, the patients in validation cohort were divided into the high-risk group and the low-risk group. Low-risk patients had statistically significantly better OS than those in the high-risk group (Log-rank *p*-value = 2.54 × 10^−6^, Figure 5). To compare the sensitivity and specificity of survival prediction, a time-dependent ROC curve analysis of this 3LMSig-based risk score model was performed. The area under the curves (AUCs) of the nomogram model in 1-, 3-, and 5-years were 0.766, 0.707, and 0.68, respectively (Figure 5), which suggested the good performance of the risk score signature.

**FIGURE 5:** The validation of 3LMSig-associated prognostic risk model.

## Discussion

Prognostic prediction of Hepatocellular carcinoma (HCC) patients has been challenging due to the complicated etiologic variables and high-level heterogeneity of HCC (Liang et al., 2020). Therefore, there is an additional need for the development of novel prognostic models, considering the limited treatment strategies for HCC. Emerging data suggest that changes in tumor lipid metabolism, including metabolite abundance and lipid metabolic product accumulation, contribute to tumor formation and local immunosuppression in the TME (Hao et al., 2019). As a result, we focused on learning more about the link between tumor lipid metabolic genes and prognosis in HCC. We seek to develop a panel of prognostic markers using molecular markers derived from tumor metabolic genes.

In this study, the public gene expression data from the TCGA-LIHC database were utilized to classify HCC patients into three molecular subtypes C1-3 based on 243 lipid metabolism-related genes. Several significant disparities in prognosis, clinicopathological characteristics, and immune and ferroptosis-related status were found across the three subtypes, especially between C1 and C3 subgroups. For example, a recently discovered cell death mechanism called ferroptosis may serve as a therapeutic biomarker for HCC. We observed C3 and C1 cluster can be classified as ferroptosis-high and ferroptosis-low groups according to the expression levels of ferroptosis-related genes. Previous research inferred the ferroptosis-high group have a worse prognosis and higher immune score (Deng et al., 2021), in line with our findings.

Then, 57 DEGs between these two subgroups were identified. GO and KEGG enrichment analysis displayed that these DEGs were closely associated functionally with lipid metabolism and tumorigenesis. Selected by machine-learning- based feature selection afterward, a prognostic risk model including 3LMSig was established. The risk model consisting of CXCL8, SLC10A1, and ADH4 was effective in predicting the prognosis of HCC patients. Moreover, the risk score calculated from the established risk model divided patients into high-risk and low-risk groups. The risk model showed that high CXCL8 expression level was associated with a bad prognosis, and high expression of SERPINC1 and ADH4 was related to better overall survival. The ROC curve analysis confirmed the moderate discriminatory accuracy of the model. According to findings, the lipid metabolism-related signature has prognostic significance for HCC. Previous research reported that SLC10A1 (solute carrier family 10 member 1) can inhibit the Warburg effect to suppress HCC tumor growth (Lu et al., 2020). ADH4 (Alcohol dehydrogenase 4), a member of the ADH family, metabolizes a wide variety of substrates including ethanol and retinol (Wei et al., 2012). CXCL8 is a promising prospective prognostic and tumor TME-related cluster (Zhu et al., 2020).

The advantage of this study is that we have identified a prognostic feature by 3LMSig that predicts 1-, 3-, and 5- year survival with relatively high AUC. However, there are limitations to this initial work. Some of the findings from this study could not be explained satisfactorily given our current limited knowledge of cancer biology. Moreover, independent studies are warranted to replicate our findings.

In summary, our study divided HCC patients into three lipid metabolism-related molecular subtypes with different prognoses and other molecular features. Then, a risk model with a good performance in prognostic prediction was built using the TCGA dataset. This model can be used as an independent prognostic evaluation index for HCC patients. Our work shed lighter on the possible significance of the lipid metabolism-associated model in stratifying patient prognosis and its feasibility to guide therapeutic selection.

## Data Availability

Publicly available datasets were analyzed in this study. The names of the repository/repositories and accession number(s) can be found in the article/supplementary material.
